The article "A Machine Learning Model for Early Prediction and Detection of Sepsis in Intensive Care Unit Patients" was retracted in 2023. Reasons: signs of a paper mill; suspected computer-generated content; unreliable results or conclusions; lack of ethics approval or compliance.

# A Machine Learning Model for Early Prediction and Detection of Sepsis in Intensive Care Unit Patients

**DOI:** 10.1155/2022/9263391

**Published:** 2022-03-26

**Authors:** Yash Veer Singh, Pushpendra Singh, Shadab Khan, Ram Sewak Singh

**Affiliations:** ^1^Department of Information Technology, ABES Engineering College, Ghaziabad (UP) 201009, India; ^2^Department of Information Technology, Raj Kumar Goel Institute of Technology, Ghaziabad (UP) 101003, India; ^3^Department of Computer Science & Engineering, Sunder Deep Engineering College, Ghaziabad (UP) 201002, India; ^4^Department of Electronics and Communication,School of Electrical Engineering and Computing, Adama Science and Technology University, Adama, Ethiopia

## Abstract

In today's scenario, sepsis is impacting millions of patients in the intensive care unit due to the fact that the mortality rate is increased exponentially and has become a major challenge in the field of healthcare. Such peoples require determinant care which increases the cost of the treatment by using a large number of resources because of the nonavailability of the resources. The treatment of sepsis is available in the early state, but treatment is not started at the right time, and then it converts to the advanced level of sepsis and increases the fatalities. Thus, an intensive analysis is required to detect and identify sepsis at the early stage. There are some models available that work based on the manual score and based on only the biomark features, but these are not fully automated. Some machine learning-based models are also available, which can reduce the mortality rate, but accuracy is not up to date. This paper proposes a machine learning model for early detecting and predicting sepsis in intensive care unit patients. Various models, random forest (RF), linear regression (LR), support vector machine (SVM), naive Bayes (NB), ensemble (of SVM, RF, NB, and LR), XGBoost, and proposed ensemble (of SVM, RF, NB, LR, and XGBoost), are simulated by using the collected data from intensive care unit patient's database that is based on the clinical laboratory values and vital signs. The performance of the models is evaluated by considering the same datasets. The balanced accuracy of RF, LR, SVM, NB, ensemble (of SVM, RF, NB, and LR), XGBoost, and proposed ensemble (of SVM, RF, NB, LR, and XGBoost) is 0.90, 0.73, 0.93, 0.74, 0.94, 0.95, and 0.96, respectively. It is also evident from the experimental results that the proposed ensemble model performs well as compared to the other models.

## 1. Introduction

Sepsis is one of the leading life-threatening diseases that rapidly infect the human system in terms of damage to the tissues. Generally, sepsis infects the organs of the human being and affects the infection-fighting process of the human body because the body's functionality works poorly and abnormally. The septic shock may occur due to the progress of the sepsis. Sepsis directly decreases the blood pressure and can create a serious problem due to the fact that various severe organ problems may occur which increase mortality. On-time detection of sepsis may be treated by the doctors using antibiotics and intravenous fluids [1]. Sepsis is the main cause of increases in mortality rate in the emergency ward. Its presence in the human body causes tissue damage and multiple organ failure. The human being immune system acts as a gatekeeper; it prevents the entry of bacteria, viruses, and so on into the body. Sepsis damages the human being's immune system, and it stops fighting against the invader. Doctors suggest that some antibiotics and antivirals protect the immune system, but sometimes they fail to recognize the appropriate antibiotic, and the selection of wrong antibiotics leads to blood poisoning in the human body and developing the severe risk of sepsis. In its early stage, the identification of sepsis is an onerous task. The definition of sepsis is changed in recent years; the new definition of sepsis provides more understanding about the occurrence of diseases and the selection of appropriate antibiotics [2].

In sepsis, various types of scoring systems are used to identify the types of sepsis and the level of risk among the patients in ICU. Sepsis is diagnosed in the presence of signs and symptoms, not based on infection, because not all infections indicate the presence of sepsis. The scoring system identifies the infection related to sepsis. Some commonly used sepsis-related ICU scoring systems [3] mentioned are quick sequential organ failure assessment (qSOFA), simplified acute physiology score (SAPS), organ dysfunction and infection system (ODIN), therapeutic intervention scoring system (TISS), acute physiology and chronic health evaluation (APACHE), modified early warning score (MEWS), early warning score (EWS), Glasgow coma scale (GCS), and mortality prediction model (MPM); SOFA is the most popular scoring system used in ICU to analyze patient's health. The first score is calculated individually for each organ; then, an aggregate is calculated to assess the final score [4]. Six physiological systems are used to calculate the final score, and they are the respiratory system, hepatic system, neurological system, cardiovascular system, coagulation system, and renal system. The scale values 0 to 4 are associated with every organ [5], scale value 0 indicates normal health, and scale value 4 indicates a high degree of dysfunction. A low score indicates good health, and a high score indicates critical health. The SOFA score is calculated during patients' ICU to stay for every 24 hours.

The machine learning-based framework could help to reduce the distance between patients and doctors because many deaths in the emergency ward are caused by human errors. The framework relies on machine learning to significantly reduce the mortality rate through smart warnings and preventive techniques [6]. Sometimes sign and doctors cannot easily recognize symptoms. Thus, the machine learning model is learning the sign and past history from previous patients' electronic databases. The machine learning-based models learn lots of data in less amount of time. The machine learning-based models automatically learn data from the database, reducing the manual intervention cost and time. Manual learning is a late process to diagnose infection and delays in selecting treatment. The manual treatment process is based on the knowledge of the doctor and by using some scoring system, whereas automatic learning is based on computational intelligence like machine learning, deep learning, and artificial intelligence [7]. It helps recognize diseases and diagnosis, selection of antibiotics, the discovery of drugs, vast collection of past medical data, smart health monitor, and so on. Automatic learning uses supervised learning (classification and regression) or unsupervised learning (clustering and association) techniques to learn the problem pattern and identify the correct label. Some popular machine learning techniques currently used in the hospital environment are support vector machine (SVM), random forest (RF), naive Bayes classifier (NB), linear regression (LR), and convolutional neural networks. Automatic learning reduced the treatment cost, staff, doctors, resources, length of stay in health infirmary, mortality rate, and so on in the modern hospitalization system. By considering the above scenarios, this paper proposes a machine learning model for early detecting and predicting sepsis in intensive care unit patients. Various models, RF, LR, SVM, NB, ensemble (of SVM, RF, NB, and LR), XGBoost, and proposed ensemble, are simulated by using the collected data from the intensive care unit patient's database on the clinical laboratory values and vital signs.

### 1.1. Contribution

This paper proposes a machine learning model for early prediction and detection of sepsis in intensive care unit patients. First of all, the missing data are collected by using the imputation process and applying matrix factorization to improve the model's performance. Secondly, different models like SVM, RF, NB, LR, and XGBoost are developed using various machine learning packages. Then, the proposed ensemble method is proposed, which combines SVM, RF, NB, LR, and XGBoost. The proposed method delivered a good classification that improves the proposed performance.

The rest of the paper is structured as follows. In Section 2, the literature review of the existing techniques is discussed. Sections 3 and 4 discuss the system model and the proposed methodology, respectively. The experiment results and discussion are given in Section 5, and finally, the paper is concluded in Section 6.

## 2. Literature Review

Generally, sepsis is identified and detected using pathology reports, physiological, biomedical signals, and so on in an ICU. The literature review of the existing studies is given as follows to identify patients with sepsis. Liu et al. proposed a multilayer approach to prognosticate patients' risk of readmission within the thirty days of discharge from the emergency ward [8]. In this work, the authors used a large set of real-world patient data on Microsoft azure for the research platform. The first attempt is to learn the network structure by using the constraint-based method, score-based method, and hybrid approach, the second is the parameter learning approach to compute probability distribution function, and the third approach is generating a set of intervention rules. Further, implement three different types of structure learning algorithms, hill-climbing, grow shrink, and hybrid, and compare their results with a baseline implementation using logistic regression. Nedee et al. proposed machine learning models that offer an automated procedure that yields steady and quick recognition of the different levels of sepsis [9]. In this work, authors assess temporal models, such as bidirectional long-short-term memory (LSTM) network and recurrent neural network (RNN), and compare the prediction performance to identify positive blood cultures. The dataset was collected from the MIMIC-III database and Ghent University Hospital for the evaluation of models for both blood culture detection and sepsis prediction, and feature was selected from both datasets for the implementation of models python TensorFlow framework.

Calsavara et al. discussed two different approaches for identifying sepsis; that is, the first models provide a prediction of short-term risk due to sepsis [10]. In this model, patients' medical parameters are collected in a short time window. In the second model prediction of long-term sepsis, the prediction was explored, which aims to collect patient data from a longer time period. Here, 33 patients are considered with a mean age of 49, out of which 19% were female, and the rest were male patients. LOS in the emergency ward, ICU scoring values, antibiotics, antivirals, age, family history for hereditary diseases, and so on were the factors associated with short- and long-term sepsis. After discharge from ICU, 24 hours was chosen to continuously observe patients who suffer from sepsis. Identification of long-term sepsis requires a more complex framework and appropriate medical parameters. Burdick et al. designed a system that helps early diagnosis of different levels of sepsis [11]. These studies evaluate the outcome of the ML algorithm for sepsis prediction and detection. Dataset was collected from Cabell Huntington Hospital (CHH). This framework helps analyze clinical patient data before and after hospital admission. Calvert et al. discussed machine learning-based sepsis diagnostic techniques using the electronic health record (EHR) data from past patients [12]. In this work, a min set of clinical variables are used for model training; the min set of variables reduced the complexity of the proposed framework as well as implementation cost and time. The machine learning techniques reduced the hospital mortality rate compared to the existing approaches used in hospital premises. Clinical variables help calculate scores to determine which patients are at the high-risk level of sepsis. The machine learning-based diagnostic (MLD) model could be beneficial to prioritize the patients according to the pathological scoring system. It provides an overview of several ML techniques for the identification of sepsis.

Fang et al. discussed a method for e-health ultrasonic diagnostic system for cardiac insufficiency and neuronal regulation in patients with sepsis using an image reconstruction algorithm [13]. Shashikumar et al. discussed a method called DeepAISE, which defines a model for early prediction of sepsis using an interpretable and recurrent neural survival [14]. This method learns predictive features by considering clinical risk factors that maximize the data likelihood of observed time to septic events. Liu et al. discussed a method called HeMA, where a hierarchically enriched machine learning approach for managing false alarms is introduced in real-time [15]. Here, a two-stage framework is developed; in the first stage, a machine learning model using statistical and particularly Kolmogorov–Smirnov tests is paired, whereas the second stage predicts whether a patient would develop sepsis. Nesaragi et al. discussed a tensor learning of pointwise mutual information from electronic health records (HER) data for early sepsis prediction [16]. The EHR data of clinical covariates capture both linear relationships and nonlinear correlation for the early sepsis prediction. Here, the statistics of pairwise association for each hour-covariate pair within the EHR data are labeled using pointwise mutual information (PMI) matrix. Rafiei et al. discussed a method for early prediction of sepsis using a fully connected LSTM-CNN model called SSP [17]. This method works in two modes; firstly, it uses demographic data and vital signs, and secondly, it uses laboratory test results and demographic data and vital signs. It uses the PhysioNet/CinC Challenge dataset, which includes the records of 40,366 patients admitted to the ICU. Yao et al. discussed a probabilistic modeling approach for interpretable inference and prediction with data for sepsis diagnosis [18]. This method uses three aspects: first, evidence acquisition based on likelihood analysis, second, probabilistic rule-based inference, and third, optimization using machine learning algorithms. It uses 4-fold cross-validation to train and validate classifiers established by the new approach and alternative ones.

Kuo et al. developed a method using an artificial neural network for early detection of sepsis with intentionally preserved highly missing real-world data for simulating clinical situation [19]. It is built with a low percentage of missing values and a high rate of missing and erroneous data to enable prediction under missing, noisy, and erroneous inputs, as in the actual clinical situation. Zhang et al. discussed an interpretable deep-learning model for early prediction of sepsis in the emergency department [20]. It uses an LSTM-based model that captures irregular time intervals with time encodings, and the model is the interpretation that enables real-world clinical applications. Kok et al. discussed the automated prediction of sepsis using a temporal convolutional network [21]. It is robust with high accuracy and precision and has the potential to be used as a tool for the prediction of sepsis in hospitals.

Chaudhary et al. discussed outcome prediction of patients for different stages of sepsis using machine learning models [22]. The paper has discussed many machine learning (ML) models that can help to predict the current stage of sepsis using existing clinical measurements like clinical laboratory test values and crucial signs in which patients are at high risk. Goh et al. discussed an artificial intelligence-based method for sepsis early prediction and diagnosis using unstructured data in healthcare called the SERA algorithm [6]. This method uses both structured data and unstructured clinical notes to predict and diagnose sepsis. Mitra et al. discussed a sepsis prediction and required signs-based approach on ranking in intensive care unit patients [23]. It uses multiple rule-based and ML models for sepsis detection and first neural network detection and prediction results on three categories of sepsis. It uses the retrospective medical information mart for intensive care (MIMIC) III dataset, restricted to intensive care unit (ICU) patients. Desautels et al. discussed the prediction of sepsis in the intensive care unit with minimal electronic health record data using a machine learning approach [24]. This method uses multivariable combinations of easily obtained patient data (vitals, peripheral capillary oxygen saturation, Glasgow Coma Score, and age), to predict sepsis using the retrospective MIMIC-III dataset, restricted to ICU patients. Papers [25–28] discussed various ensemble schemes based on language function analysis, web page classification, automated breast cancer diagnosis, text sentiment classification, text classification, and feature engineering for text genre classification.

## 3. System Model

This section will discuss the process of dataset exploration, data cleaning and data extraction, feature selection, model building, and machine learning classification models. In the experimental setup, we use the hardware configuration as Intel Core-i7 CPU and 8 GB RAM, whereas in software configuration, we use Windows 10 operating system, python 3.0 as the programming language, anaconda as python distribution, and various python libraries, namely, Pandas, Matplotlib, NumPy, iPython, Seaborn, Jupyter Notebook, and scikit-learn. In this work, the publicly available patient's dataset “Skaraborg Hospital” is used, collected between 2011 and 2012. It has 1572 sepsis patient records with respect to 67.3 years of age on average. Additionally, out of 1572 sepsis patient records, 55.6% are male patients, and 44.4% are female patients. The training set uses 1257 patient records, whereas the 315 records are used for testing purposes. This dataset contains the data like antibiotics to treat disease, sepsis-2 criteria, sepsis-3 criteria, vital signs, positive blood culture, survival data, hospital length of stay, and so on.

In the process of data cleaning and data extraction first, check the format of the data and these attributes. The available data are in the comma-separated values (CSV) file. The available data contains various features, age, gender, and so on, which are converted into dummy features as numeric features, which can be handled easily. After that, the processing of the missing data values is handled; it directly affects the performance of the model. The data imputation technique is used for generating the missing data, that is, the average mean, and it helps in the performance improvement. The kernel density estimation is used for data exploration in the process of outlier detection. After completing the above process, a separate file is created for the sepsis dataset, and these records are divided into training and testing using various python libraries. Then the machine learning model is trained using the sepsis dataset. Further, some useful tools to explore more data are applied, which make smarter decisions. Moreover, import Seaborn Python library to plot histogram and pie chart distributions to analyze the hidden data.

The important interaction between features is very important in the prediction model because some features depend on the existence of other features; if the interaction between features is not handled, then prediction cannot have expressed completely. At a particular point in time, additional feature selection mitigates the precision of the models; this is known as the curse of dimensionality. To come out from these advantages, applied dimensionality reduction using principal component analysis (PCA) is used to describe the data efficiently and also allow to elect more features. The major benefits of using dimensionality reduction are mitigating the model complexity and avoiding overfitting. Feature selection and feature extraction are considered two major components of dimensionality reduction. In feature selection, select the original features that are useful to boost the productivity of models. In feature extraction, extract the useful information from the original feature set to build a new subsample dataset with fewer variables. Feature extraction can help improve computational efficiency and enhance the predictive power of ML models by reducing the curse of dimensionality.

The feature selection and model building, first of all, select the comprehensive set of features, that is, good for the measurement, and predict and identify the good results. For example, classify sex value 1 for male and 0 for female; age, heart rate, blood pressure, RR, procalcitonin, temperature, platelet count, WBC count, SOFA score, SBP, DBP, mean arterial pressure (MAP: it is a combination of SBP and DBP), SIRS criteria, oxygen saturation (SpO2), hemoglobin, partial pressure of oxygen (PaO2), creatinine, total time in hospital, Glasgow coma scale (GCS), c-reactive protein serum, and p-lactate were sampled and employed in the predictive models. In this process, we followed the instructions provided by the “surviving sepsis campaign and mayo clinic” administration of sepsis and septic shock, and based on this knowledge, it is easy to pick the inclusion and exclusion criteria to include and exclude the parameters [29].

In this work, the backward elimination process is used for the feature selection in the process of building the model. This process removes those features that do not significantly affect the dependable variables. Initially, it considers all the independent variables and then removes those variables which are not significant using the statistical method. In the process, a significance level is selected to stay in the model, which is defined as 0.05. Then, fit the whole model with all the possible independent/predictors variables. The predictor variables are chosen that have the highest *p*-value (value of the particular feature). If the *p*-value of any particular feature is greater than the defined significance level value, then remove that predictors variable; otherwise, stop the process, and the model is ready. After that, rebuild and fit the model with the remaining variables. This process considers the most significant features and removes the unnecessary features which increase the complexity of the model.

Now, we will discuss the various classifiers which are used to detect and predict sepsis. A classifier is an algorithm that machines use to categorize data. The ultimate proposed model of the selected classifier in machine learning is a classification model. The classifier is used to train the model, and the model is then used to classify the available data. The training datasets are provided to supervised and semisupervised classifiers, which teach them how to categorize data into specified categories. Below machine learning classifiers and their ensembles are used in this work, namely, support vector machine, naive Bayes, random forest, logistic regression, and XGBoost. The dataset was used to select and test supervised learning classifiers. The machine learning algorithms that were used in this study are briefly described here.

### 3.1. Support Vector Machine (SVM)

SVM is one of the most effective classifiers, which has some sort of linearity. It has good mathematical intuition behind the SVM and is capable of handling some situations where nonlinearity is present by using a nonlinear basis function. This type of function is called kernel function. SVM intelligently stops overfitting and works more attributes or features without more computation [30]. The output is the optimal hyperplane if the training data labeled are given to the SVM algorithm, and a new example is given for the classification. The hyperplane is dividing the plane where each class is placed in either side. The line is treated as a hyperplane for two-dimensional planes; similarly, for three-dimensional spaces, the plane is treated as a hyperplane. When the line is not dividing the plane, then transformation is done to the next higher dimension. If that dimension separates the class, then it transfers to the next higher dimension. Similarly, this transformation is done repeatedly until it divides the class separately. If the data points are overlapping, we cannot get the linear line. To correctly divide the classes, we need a nonlinear line. For this, the support vector machine uses tuning parameters. Regularization parameter and gamma are used for this purpose. If we change this value, we get a nonlinear classification line. The kernel is used as one of the tuning parameters. It transfers the problem into linear algebra.

### 3.2. Naive Bayes Classifier (NB)

The naive Bayes model selects the hypothesis (*h*) based on some prior knowledge about the data points. It evaluated the probability value of *h* using prior knowledge. It is based on conditional probability, and it finds out posterior probability from prior probability. When we calculated the posterior probability for various hypotheses, we selected the one which contributes to maximum probability [31]. Naive Bayes is used for classification problems. It stores the probabilities of every class present in the dataset and then learns the model. It uses class probability and conditional probability. In the training dataset, it calculates class probability, and conditional probability is calculated for each input value over a given class value. It is very fast to learn from the training data because only class and input probability are calculated. Class probability is calculated as the ratio of the frequency of each class to a total number of instances. The conditional probability is calculated as the ratio attribute frequency value of a given class to the frequency of instance of that class. It also extends to real value by considering Gaussian distribution.

### 3.3. Random Forest (RF)

This model is an ensemble of the set of decision trees which is trained in a parallel manner [32]. The RF uses an augmentation of the decision tree classifier with respect to a set of trees. RF ensemble is widely used in various environments and industries because of its simplicity, parallelized working, and strong outliers with distorted data. It also provides good accuracy because it uses the week estimators while fine-tuning. The main reason to opt out of the random forest for the prediction and determine the sepsis works well during underfitting the enormous dataset. The whole dataset is divided into 80 : 20 ratios for training and testing point of view, and RandomForestClassifier from sklearn python library is applied to check the performance of the model and fine-tune the parameters of the random forest. Pass all the test set samples to the randomly created trees to predict the new samples on the trained set. Each tree in the forest produces a different outcome on the same test features. The procedure is repeated for each test feature. Ultimate prediction is selected based on the majority of voting, and the tree that gets more votes in the forest is considered as the final classifier.

### 3.4. Logistic Regression (LR)

This method is based on the supervised machine learning classifier and is widely used for analyzing laboratory data [33]. It is an extremely interpretable model which is appropriate for the baseline model in terms of comparisons of existing models. This method uses the binary variable (0 and 1) as dependent variables to predict whether the patient is suffering from sepsis or the patient is not suffering from sepsis. There is a package in python, namely, the linear model LR, which can be imported to build the model. The whole dataset is divided into 80 : 20 ratios for training and testing point of view, and a 10-fold cross-validation technique is applied. Furthermore, GridSearchCV has been used to fine-tune the parameter for increasing the model efficiency. The equation representation of LR is much similar to linear regression. In a 2D graph, the *x*-axis is considered a set of independent features. The *y*-axis is considered the target variable or dependent feature required for the prediction.

### 3.5. XGBoost

This subsection will show the effectiveness of the XGBoost machine learning model, which is used to predict sepsis. This method is also known as the eXtreme Gradient Boosting method. Here, boosting is an ensemble approach where new models are combined to correct the errors based on the old models [34] by using tree learning and linear model solver algorithms. It is a faster method because of its nature of parallel computation, and the performance of the model can be improved by built-in cross-validation and fine-tuning the parameters. Regression and classification are two main objective functions that encourage us to use the XGBoost model for prediction. Compared to other machine learning algorithms, it provides a better solution for classifying models because it supports numerous boosting parameters. The main motives to choose XGBoost include efficiency, ease to use, accuracy, feasibility, built-in cross-validation, and a wide range of tuning parameters available. The idea of boosting is an algorithm that qualifies to fit various weak classifiers to reweighted versions of the training data and generate final results by combining the results of the predecessor classifier. A set of weak learners is transformed into strong learners by boosting technique [35]. The boosting algorithm is mainly classified into three types: AdaBoost (Adaptive Boosting), Gradient Boosting, and XGBoosting. When we used boosting technique, all samples in the dataset were allotted with a score that notifies how difficult they are to classify. In each of the following iterations, the algorithm pays more awareness to the cases that were wrongly classified previously. One or more weak classifier is combined to form a final classifier with no error.

## 4. Proposed Methodology

In this work, machine learning models for the prediction of different stages of sepsis are proposed. Here, a frame of the problem of early prediction and detection of different stages of sepsis as a classification problem is developed. The objective is to continuously update the predicted probability that the encounter will result in sepsis using all accessible patients' information up till that time. In the existing machine learning model, we introduced some new mechanisms like 10-fold cross-validation, hyperparameter tuning, boosting parameters, creating parameter candidates to find the most accurate parameters for the specific model, and conducting GridSearchCV for parameter tuning to find out the parameters that achieved the highest score. At each fold, we split the training dataset and test with a different set of data and calculated the performance metrics at each fold to evaluate the accuracy of the models. The experimental workflow of the proposed method is shown in Figure 1. The first step is the dataset loader; after performing the data imputation, data cleaning, data preprocessing, data transformation, feature selection, and feature extraction, the details of all data processing and data visualization techniques were discussed in the previous section. For cross-validation of the training dataset, we exploited k-fold cross-validation procedures. We choose *k*=10 to split the dataset into 10-fold, out of which ninefold is employed for training, and onefold is used in favour of the test set to compare the training dataset on the test dataset at each fold; this operation is recurring for the whole split. After cross-validation, we applied parameters tuning, out of which select the best parameter for the model tuning. After generating the optimal parameter model, classify the beat label to predict patients who suffer from sepsis and those who do not suffer from sepsis. Further, they were classified into two groups: patients die or survive in ICU. We compared the performance of all the models based on the obtained results from each model and found out which models give a more accurate result for the prediction of sepsis.

Ensemble learning model: this section outlines the implementation of the ensemble model. It uses multiple ML models to make satisfactory prediction results on a dataset. An ensemble model works by training distinct models on a dataset and having each classification model makes predictions individually; the obtained results of these models are then incorporated into a single model to make a final prediction. Every machine learning model has some pros and cons. Some models work well on a particular dataset, and some do not. So what the ensemble learning model is doing is that it combines the best features of each model in order to make precise predictions. The three most popular techniques are generally used to combine the obtained results from distinct models into a single one; they are as follows.

(i) Bagging-based ensemble learning: combine the results of multiple models to get a generalized result. Bootstrapping sampling technique is used to create different observations from the training dataset. Bagging reduced the variance of the model.

(ii) Boosting-based ensemble learning: create several models; every single model learns to fix the prediction errors of a preceding model. Boosting technique based on the sequential learning approach. Each model in a chain is connected to the other in cascading fashion. The output of one model becomes the input of another subsequent model. It works on the principle of a weak classifier; all the weak classifier combines to form a strong classifier in order to reduce the model errors, reduce the bias and boost the performance of the models. Some popular boosting techniques have been used by researchers in recent years, such as AdaBoost, CatBoost, random forest estimators, and Gradient Boosting [36].

(iii) Voting-based ensemble learning: establish multiple models, and then elementary statistics are used to integrate the prophecy of the models. It is one of the most straightforward ensemble learning techniques in which predictions from multiple models are combined based on the voting. In this section, we mainly focused on voting-based ensemble learning. There are three most popular voting methods used in voting-based ensemble learning:

(i) Majority voting: majority voting is sometimes also referred to as plurality voting. Forecast the class label “*u*” via majority (plurality) voting from every single classifier. Here, we apply the mode method to find out the highest occurrence of frequency. For example, if we select classifier (1) which classify as *C*(0), classifier (2) which classify as *C*(1), similarly classifier (3) which classify as *C*(0), by taking mode of *C*(0) that occurs twice, so via the majority vote model classifies the pattern as the class label “*C*(0).”
  (1) $$\begin{array}{c} u=\text{mode}\left\{C1\left(x\right),C2\left(x\right),C3\left(x\right)\ldots \ldots \ldots Cm\left(x\right)\right\}. \end{array}$$
(ii) Weighted majority vote: weight is assigned to each classifier. For example, we select three classifiers 1 to 3 and assign weight (1, 0.2, and 1(. Here, we classify the class with max weight.
(iii) Soft voting: compute the average probabilities for each classifier and win the class that got the highest probabilities value. In the proposed work, we ensemble LR, SVM, RF, NB, and XGBoost classification models as shown in Figure 2 to build the ensemble learning model.

To build the ensemble learning models, the following steps need to be followed.

**Step 1 .**

Load the CSV format dataset using the CSV module.

**Step 2 .**

Import python scikit-learn library.

**Step 3 .**

Divide the whole dataset into test and train records by using “sk learn.model_selection import train_test_split” and pass the value to the train_test_split function parameters such as test_size, train_size, and random_state.

**Step 4 .**

Select the classifier models to import the following python libraries: from sklearn “import model_selection,” from sklearn.svm “import *SVC*,” from sk learn.naive_bayes “import GaussianNB,” from sk learn.ensemble “import RandomForestClassifier,” and from sk learn.linear_model “import LogisticRegression.”

**Step 5 .**

*x*_train is a standalone factor in training records and *y*_train is the target factors.

**Step 6 .**

To implement the voting-based ensemble learning techniques, import the following python libraries: from sklearn.ensemble import VotingClassifier, sklearn.ensemble “import VotingClassifier” and from mlxtend.classifier “import EnsembleVoteClassifier.”

**Step 7 .**

To enhance the performance of the ensemble model, apply the test on different parameters and cross-validation and tune the hyperparameter.

**Step 8 .**

There are three steps for combining the predictions of classification models, which are given as follows: firstly, a base learner's library is selected for generating the predictions, secondly, a metalearner is elected, which helps in the learning process of “how to best combine these elected predictions,” and finally, a method for dividing the data of training is chosen between the base learners and the metalearner.

**Step 9 .**

Select the majority voting method and associate the predictions obtained from each one of the classification models into a final prediction.

**Step 10 .**

Compute the ensemble learning models' performance metrics; repeat Step 6 until we get the best results from the ensemble model.

## 5. Simulation Results and Analysis

In this work, a prediction and detection model is formulated to predict and classify the onset of distinct stages of sepsis before or after its occurrence by using machine learning classifiers models. Here, various experiments, including data cleaning, imputation techniques, feature selection, feature extraction training, parameters tuning, parameters optimization, GridSearchCV, cross-validation, and testing phases for our model, are performed. The publicly available sepsis patient's intensive treatment unit (ICU) datasets are used to perform these experiments. We have also evaluated our results in comparison with state-of-the-art methods discussed in the literature review. In this section, we will also introduce the evaluation metrics required for the analysis of the ML model performance and train for the prediction and detection of different conditions of sepsis. In this work, five different classification models are considered for checking the performance, that is, support vector machine (SVM), random forest (RF), naive Bayes classifier (NB), linear regression (LR), and XGBoost. An ensemble model (of SVM, RF, NB, LR, and XGBoost) is also considered for evaluating the performance, which is based on performance metrics that are selected from the various existing binary classification models.

The evaluation metrics are helpful tools to analyze the performance of various machine learning models. It could help to select which model is performed best and which one performed worst for a particular type of problem. There are several machine learning metrics that exist for the performance analysis of classification and regression models. The tedious task is how to find suitable evaluation metrics for the defined problem. Some of the metrics are given as follows: the confusion matrix is one of the best metrics that can help analyze the classification performance of the existing and the proposed models. The confusion matrix can be categorized into four different categories based on the correctly predicted and confusing term, that is, true positives (TP), true negatives (TN), false positives (FP), and false negatives (FN). The first two are used to observe the correctly predicted classification, and the last two define the confusion in the matrix. The first TP is the classifier that predicted “sepsis” and defined the patients who have sepsis disease (*y*_true=1, *y*_pred=1). The second TN classifier predicted “no sepsis” and defined the patients who do not have sepsis disease (*y*_true=0, *y*_pred=0). The third FP classifiers predicted “sepsis” and defined patients who do not actually have sepsis disease (*y*_true=0, *y*_pred=1), and the fourth FN classifier predicted “no sepsis” and defined patients who actually do have the sepsis disease (*y*_true=1, *y*_pred=0). Other metrics are given as follows.

Accuracy: it is the percentage of total items classified correctly, which represents the percentage of patients whose labels were properly recognized. The confusion matrix evaluation of accuracy is as follows:

(2) $$\begin{array}{c} \text{accuracy}=\frac{\left(\text{TP}+\text{TN}\right)}{\left(\text{TP}+\text{FP}+\text{TN}+\text{FN}\right)}. \end{array}$$

Precision: it defines the percentage of patients who were diagnosed as having infection are actually correct. The confusion matrix evaluation of precision is as follows:

(3) $$\begin{array}{c} \text{precision}=\frac{\left(\text{TP}\right)}{\left(\text{TP}+\text{FP}\right)}. \end{array}$$

Sensitivity/recall: it is an evaluation metric in terms of percentage where it confirms that the patent has sepsis that is diagnosed by the model properly. The sensitivity and specificity are dependent on each other if the sensitivity value of the predicted class increases; it means that the specificity of the predicting class decreases. The higher the sensitivity, the more the predictive power of the model. When precision is equal to recall, this situation is known as the breakeven point. The confusion matrix evaluation of sensitivity is as follows:

(4) $$\begin{array}{c} \text{sensitivity}=\frac{\left(\text{TP}\right)}{\left(\text{TP}+\text{FN}\right)}. \end{array}$$

Specificity: the test finds that the parent is healthy. The confusion matrix evaluation of specificity is as follows:

(5) $$\begin{array}{c} \text{specificity}=\frac{\left(\text{TN}\right)}{\left(\text{TN}+\text{FP}\right)}. \end{array}$$

F1 measure: it is the combination of recall and precision. From (2) and (3), evaluation of the F1 measure is shown as follows:

(6) $$\begin{array}{c} F1\text{ score}=\frac{2*\text{precision}*\text{recall}}{\text{precision}+\text{recall}}. \end{array}$$

The area under the receiver operating characteristics (AUROC) represents the receiver operating characteristic (ROC) for the false positive rate (FPR) in terms of probability curve and for the true positive rate (TPR) in terms of quantifying the separability and represents the *x*-axis and *y*-axis, respectively. The ROC plot is grounded on a pair of fundamental assessments, that is, specificity and sensitivity. The specificity is a performance gauge of the entire negative portion of records, whereas sensitivity is a performance gauge of the entire positive portion.

The machine learning models have been trained and tested on the sepsis patient's dataset. This dataset contains a total of 1572 patients, out of which 1257 patients were selected for the training dataset and 315 patients for the test dataset. From the available vital sign, samples were collected from the human body, clinical measurements, and pathology reports on the basis of the preliminary examination. The exploit age, gender, body temperature, RR, HR, SBP, DBP, positive blood culture, MAP, Lactate, and WBC were the features selected for the model training. Along with the mentioned list, we use SIRS and SOFA scores to recognize the severity of bacterial infection. We decided to restrict the selected variables and to keep just the ones that are measured routinely and that are not directly related to sepsis are excluded. A detailed analysis of the relationships between the measured variables when the outcome variable is removed from the analysis is beyond the remit of the current brief paper. Only adult patients are considered in this study. We will account for our outcomes in two steps: firstly, associate the achievement of all the mentioned models, and subsequently, we will pick the superior model and then compare the attained results of the superior model with the other machine learning existing model for recognition of sepsis [37] and the routinely available screening scoring systems. We ran five prediction models using a machine learning method. Out of the 5 models, the highest AUC achieved is 0.96, the lowest AUC achieved is 0.74, and the average AUC of 0.88 is performed to identify different sepsis.

Figure 3 shows the accuracy, precision, recall, specificity, F1 score, and AUC of the various existing and proposed models. Additionally, the classification performance of machine learning models for the prediction and detection of sepsis is demonstrated in Tables 1 and 2.  Table 1 shows the comparison of the proposed framework and the results of different existing machine learning techniques in terms of their accuracy, precision, recall, specificity, F1 score, and AUC to identify sepsis. The proposed ensemble model of SVM, RF, NB, LR, and XGBoost with 10-fold cross-validation and hyperparameter tuning for prognostic of sepsis achieved the highest AUC. The proposed ensemble model's performance is superior to the LR, NB, RF, SVM, and XGBoost and voting ensemble learning classifier (which is the combination of LR, NB, RF, SVM, and XGBoost) in terms of predictive power for the recognition of sepsis. The balanced accuracy is computed by fetching the average positive recall and negative recall from both classes. It balanced the values obtained from both classes.

The balanced accuracy of random forest (RF) model, linear regression (LR) model, support vector machine (SVM) model, naive Bayes classifier (NB), ensemble model (of SVM, RF, NB, and LR), XGBoost, and proposed ensemble model (of SVM, RF, NB, LR, and XGBoost) is 0.90, 0.73, 0.93, 0.74, 0.94, 0.95, and 0.96, respectively. From the obtained experimental results, we conclude that the proposed method demonstrates some noteworthy improvement of the new machine learning framework for the precise prediction of different stages of sepsis. We successfully established a model for differentiation among the healthy and the unhealthy patients based on the clinical measurements and vital signs. The promising results encourage that the established methodology may be helpful in the hospital environment.

Table 2 shows that the AUC results for the proposed ensemble model (of SVM, RF, NB, LR, and XGBoost), Chaudhary et al. [22], Mitra and Ashraf [23], Desautels et al. [24], and Onan et al. [25] with the publicly available datasets Skaraborg Hospital, Skaraborg Hospital, Clinical notes, MIMIC-III, and MIMIC-III are 0.96, 0.95, 0.94, 0.89, and 0.74, respectively. The proposed ensemble model (of SVM, RF, NB, LR, and XGBoost) gives the highest accuracy, that is, 0.96, and the lowest is 0.74.

## 6. Conclusion

This paper proposes a machine learning model for early prediction and detection of sepsis in intensive care unit patients. First of all, the missing data are collected using the imputation process and applying matrix factorization to improve the model's performance. Secondly, different models like SVM, RF, NB, LR, and XGBoost are developed using various machine learning packages. Then, the proposed ensemble method is proposed, which combines SVM, RF, NB, LR, and XGBoost. The proposed method delivered a good classification that improves the proposed performance. This model is beneficial to the patients admitted to the intensive care unit. This work can be extended by collecting geographical patient data to visualize more signs and symptoms of patients to feed more data to the machine learning model. The medical dataset contains a lot of missing data that could degrade the model performance; it requires more advanced data imputation techniques to handle this problem.

## Figures and Tables

**Figure 1:** Experimental workflow for evaluating the performance of the various models.

**Figure 2:** The proposed ensemble learning model architecture.

**Figure 3:** Accuracy, precision, recall, specificity, F1 score, and AUC of the existing and the proposed models.

**Table 1:** Various models with the accuracy, precision, recall, specificity, F1 score, and AUC.

Models	Accuracy	Precision	Recall	Specificity	F1 score	AUC
Random forest (RF) model	0.90	0.95	0.88	0.94	0.94	0.91
Linear regression (LR) model	0.73	0.58	0.82	0.69	0.68	0.76
Support vector machine (SVM) model	0.93	0.94	0.90	0.97	0.94	0.93
Naive Bayes classifier (NB)	0.74	0.68	0.88	0.61	0.77	0.74
Ensemble model (of SVM, RF, NB, and LR)	0.94	0.90	0.93	0.89	0.91	0.94
XGBoost	0.95	0.97	0.92	0.97	0.97	0.95
Proposed ensemble model (of SVM, RF, NB, LR, and XGBoost)	0.96	0.98	0.94	0.97	0.98	0.96

**Table 2:** Various existing and proposed models with AUC.

S. no.	Methods	Datasets	AUC
1	Proposed ensemble model (of SVM, RF, NB, LR, and XGBoost)	Skaraborg Hospital	0.96
2	Chaudhary et al. (XGBoost) [22]	Skaraborg Hospital	0.95
3	Mitra and Ashraf [23]	Clinical notes	0.94
4	Desautels et al. [24]	MIMIC-III	0.89
5	Onan et al. [25]	MIMIC-III	0.74

## Data Availability

Data will be available upon request to Yash Veer Singh (yashveersingh85@gmail.com).
